# MiR-200c/FUT4 axis prevents the proliferation of colon cancer cells by downregulating the Wnt/β-catenin pathway

**DOI:** 10.1186/s12885-020-07670-y

**Published:** 2021-01-04

**Authors:** Jinchun Cong, Jian Gong, Chuanjia Yang, Zhixiu Xia, Hong Zhang

**Affiliations:** 1 Department of General Surgery, Shengjing Hospital China Medical University, No. 36 Sanhao Street, Heping District, Shenyang, 110004 China; 2 Department of Clinical Pharmacy, Shenyang Pharmaceutical University, Shenyang, 110016 China

**Keywords:** miR-200c, FUT4, Colon cancer, Wnt/β-catenin pathway

## Abstract

**Background:**

MicroRNA (miR)-200c has been widely reported to be involved in colon cancer progress. However, the mechanisms of miR-200c in regulating tumor metastasis and growth remain to be fully elucidated. This study aimed to investigate the mechanism of miR-200c targets fucosyltransferase 4 (FUT4) on the proliferation of colon cancer.

**Methods:**

The miR-200c and FUT4 mRNA levels in LoVo and SW480 cells were measured by real-time quantitative polymerase chain reaction. Further, miR-200c mimic, FUT4 siRNA and FUT4 mimic were transfected into cells, separately. Cell counting kit-8, plate colony formation and transwell assays were used to analyse the cells biological behaviour.. Immunofluorescence was used to analyse the Ki-67 expression Moreover, the Wnt/β-catenin pathway-related proteins were detected by western blots. A double luciferase experiment was performed to confirm the relationship between miR-200c and FUT4. In vivo, tumour growth and Wnt/β-catenin pathway-related proteins were also analysed.

**Results:**

In vitro, the expression of miR-200c and FUT4 were negatively correlated in LoVo and SW480 cells (correlation coefficients were − 0.9046 and − 0.9236, respectively). MiR-200c overexpression inhibited the proliferation, migration and invasion of LoVo and SW480 cells by downregulating FUT4. The Ki67-positive cells and Wnt/β-catenin signalling pathway-related proteins were reduced in the miR-200c overexpression and FUT4 silencing groups. A dual luciferase reporting system identified FUT4 as the target of miR-200c. The results in vivo were further confirmed the foundation of cells study.

**Conclusions:**

In summary, miR-200c overexpression inhibits proliferation of colon cancer targeting FUT4 to downregulate the Wnt/β-catenin pathway, which promises molecular targets to inhibit metastasis for colon cancer therapy.

**Supplementary Information:**

The online version contains supplementary material available at 10.1186/s12885-020-07670-y.

## Background

Colon cancer, a malignancy of the large intestine (colon), is a clinically highly malignant tumour of the digestive tract. Colon cancer ranks third in global gastrointestinal tumour incidence and fourth in mortality [1]. Colon cancer can cause blood in the stool, stomach pain, and changes in stool. If this disease is detected early, most patients with colon cancer can recover. However, there are more than one million new cases of colon cancer, and approximately 700,000 people die of colon cancer each year in 2013 globally [2]. Currently, the treatments for colon cancer are unsatisfactory.

MicroRNAs (miRNAs) are small endogenous noncoding RNAs that play important roles in multiple oncogenic cellular processes [3, 4]. In colon cancer, an increasing number of studies have shown that various miRNAs are involved in the process of colon cancer, including miR-200c [5, 6]. The expression of miR-200c has been found to correlate with poor prognosis of colon cancer [6]. The miR-200 family comprises 5 members, miR-200a/b/429 and miR-200c/141 [7]. Accumulating evidence suggests that miR-200c, a tumour suppressor, has low expression in colon cancer [8–11]. MiR-200c inhibitors could enhance the viability and proliferation of colorectal cancer cells (CRC), and low miR-200c expression was related to shortened survival of patients with CRC [8, 11]. However, Chen et al. [6] reported an opposite conclusion in colon cancer showing that miR-200c was highly expressed in colorectal cancer and functions by inhibiting protein tyrosine phosphatase gene expression and p53 phosphorylation. The regulation of colon cancer metastasis by miR-200c is mediated by a complex biological network [9, 10]. Therefore, the regulatory mechanism of miR-200c in colon cancer metastasis deserves further study.

Wnt/β-catenin signalling controls multiple biological phenomena in early life and adult life by regulating cell proliferation and genetic stability [12]. Studies have shown that the miR-200 family plays an important role in the regulation of cancer cell proliferation and metastasis by inhibiting Wnt/β-catenin signalling [13, 14]. Dermani et al. found that zerumbone inhibited epithelial-mesenchymal transition and cancer stem cell properties by inhibiting the Wnt/β-catenin pathway through miR-200c [15]. In this work, we investigated the effects of miR-200c on the proliferation of colon cancer. Furthermore, we studied whether its mechanism of action was related to the Wnt/β-catenin signalling pathway, searching for promising molecular targets to inhibit metastasis for colon cancer therapy.

## Methods

### Cell culture

The the human colon cancer cell lines LoVo (BNCC338601) and SW480 (BNCC288146) and human normal intestinal epithelial cell line NCM460 (BNCC353657) were obtained from the BeNa Culture Collection (www.bnbio.com, Beijing, China). These cells were derived from ATCC (Manassas, VA, USA) and have been authenticated using short tandem repeat (STR) markers. In addition, the cells have not been tested for mycoplasma contamination. Cells were cultured in RPMI-1640 (Gibco, Rockville, MD, USA) containing 10% foetal bovine serum (FBS, Sigma-Aldrich, St. Louis, MO, USA). The cells were maintained in a humidified cell incubator (Thermo Fisher Scientific, Waltham, USA) atmosphere of 5% CO_2_ at 37 °C.

### Cell groups and transfection

LoVo and SW480 cells were divided into (1) blank control group (BC): no treatment; (2) miR-200c overexpression group: cells were transfected with 100 nM miR-200c mimic (5′-TCCATCATTACCCGGCAGTA-3′) lentiviral vector; (3) fucosyltransferase 4 (FUT4) silencing group (si-FUT4): cells were transfected with 50 nM FUT4 siRNA (5′-GUUUGGAUGAACUUCGAGUTT-3′, 5′-ACUCGAAGUUCAUCCAAACTT-3′;) lentiviral vector; (4) miR-200c + FUT4 overexpression negative control group (miR-200c + NC1): cells were transfected with 100 nM miR-200c mimic and 50 nM pcDNA3.1 empty vector; (5) miR-200c + FUT4 overexpression group (miR-200c + FUT4): cells were transfected with 100 nM miR-200c mimic and 50 nM pcDNA3.1 FUT4 plasmid. Cells were transfected using Lipofectamine® 2000 (11,668,019, Invitrogen, Shanghai, China) according to the manufacturer’s protocols. In each group, there were three replicates.

LoVo and SW480 cells in logarithmic growth phase were selected for subsequent experiments. The cells were passaged 1 day before transfection and cultured in a 6-well plate. When the confluence reached 70%, transfection was performed according to the lentiviral transfection instructions. Lentiviral particles were constructed by Shanghai Jikai Biotechnology Co., Ltd. (Shanghai, China). MiR-200c mimic, FUT4 siRNA, pcDNA3.1 FUT4 and negative control lentiviral vectors were purchased from Shanghai GenePharm Pharmaceutical Technology Co., Ltd. (Shanghai, China). The expression of miR-200c and FUT4 mRNA in transfected cells was detected by real-time quantitative polymerase chain reaction (RT-qPCR) at 72 h after transfection. Each experiment was repeated three times.

### RT-qPCR

A total RNA extraction kit (A27828, MagMAX™ MiRVana™ Total RNA Isolation Kit, Thermo Fisher Scientific, Waltham, USA) was used to extract total RNA from the cells. cDNA was synthesized by a reverse transcription kit (Applied Biosystems, Waltham, MA, USA), and SYBR Green PCR Master Mix (Applied Biosystems, Foster City, CA USA) was used for RT-qPCR. The miR-200c primer was synthesized by Shanghai Shengong Biotechnology Co., Ltd. (Shanghai, China), and the reaction was performed under the following conditions (40 cycles): 95 °C for 10 min, 95 °C for 15 s, and 60 °C for 1 min. The miR-200c and FUT4 mRNA compared with the endogenous controls U6 and GAPDH, respectively, and the data were processed by the 2^-ΔΔCt^ method. The sequences of the primers were showed in Table 1.

**Table 1:** Primers used in RT-qPCR

Gene	Forward (5′-3′)	Reverse (5′-3′)
MiR-200c	CCTATGTAAACAGCCTCGACTG	CTGGCGTATCGTGAGTCG
U6	GACCTCTATGCCAACACAGT	AGTACTTGCGCTCAGGAGGA
FUT4	AAGGTCCAGGCCCACTGAAG	CAGTTCAGGTGACAGAGGCTCA
GAPDH	ATGGGGAAGGTGAAGGTCG	GGGGTCATTGATGGCAACAATA

### Double luciferase reporter assay

Target gene prediction between miR-200c and FUT4 was performed using TargetScan software (www.targetscan.org). Wild-type and mutant 3′-UTRs of FUT4 were amplified in the pGL3/luciferase vector (Promega, Madison, WI, USA) and cloned downstream of the luciferase gene. The constructed luciferase reporter plasmid (wt-FUT4 or mut-FUT4) was separately co-transfected with miR-200c or NC into LoVo and SW480 cells using Lipofectamine 2000 (Invitrogen, Thermo Fisher Scientific, China) for 24 h. The luciferase activity of the cells was detected with the dual luciferase reporter system (Promega) at 48 h after transfection according to the instructions.

### Cell counting kit (CCK)-8 assay

Cells at logarithmic growth phase were plated into 96-well plates at a density of 2 × 10^4^ cells/mL, 100 μL per well. According to the manufacturer’s instructions (G021–1-1, Nanjing Jiancheng Bioengineering Institute, China), cells viabilities were analyzed. The optical density (OD) of each well at 450 nm was measured by a microplate reader (HBA-1096A, DeTie, Shanghai, China).

### Plate colony formation assay

Logarithmic growth phase cells were digested with 0.25% trypsin and adjusted to 250 cells/mL. Cells (2 mL/well) were cultured in a 6-well plate at 37 °C and 5% CO_2_ for 2–3 weeks, and the fresh medium was added every 3 days. Methanol was used to fix the cells, and 1 ml of Giemsa working fluid (48,900, Sigma-Aldrich, Shanghai, China) was used to stain the cells for 30 min. After two washes with ultrapure water, filter paper was used to remove the water around the dish, and the cells were imaged by a camera (Eos RP, Canon, Japan).

### Transwell assay to analyse cell migration and invasion

Cell invasion experiment: After digestion, centrifugation and resuspension, the cells were adjusted to 4 × 10^5^ cells/mL. Fifty microlitres of 1640 medium containing Matrigel (1:1) without FBS was added to the transwell upper chamber and incubated at 37 °C for 1 h. Then, 100 μL of cell suspension was added to the upper compartment of the chamber, while 600 μL of complete medium containing 10% FBS was added to the lower chamber. After incubation at 37 °C and 5% CO_2_ for 24 h, the membranes were fixed with methanol for 30 min and stained with crystal violet for 15 min. The non-migrated cells in the upper layer were gently wiped with cotton swabs. The results were observed under a inverted microscope (BDS400, Aote, China) and assessed by ImageJ software 6.0 (National Institutes of Health, USA).

For the cell migration experiment, Matrigel was not required, and the other experimental steps were the same as those for the invasion experiment.

### Immunofluorescence

The cells in coverslips were treated differently as required and fixed with 4% paraformaldehyde. With 0.2% Triton X-100 cell permeabilization, the cells were blocked with 5% bovine serum albumin (BSA) and incubated in an incubator for 30 min at 37 °C. Then, the cells were incubated with primary antibodies against Ki67 (1:600, orb69312, Biorbyt, Cambridge, UK) at 4 °C overnight. After the cells were rinsed with phosphate-buffered saline (PBS), they were incubated with FITC-labelled lgG1(1:800, 11–4015-82, ThermoFisher, Shanghai, China) at 37 °C for 30 min in the dark. Subsequently, the cells were rinsed with PBS, stained with 4′,6-diamidino-2-phenylindole (DAPI, orb90525, Biorbyt, Cambridge, UK) and mounted with glycerol. The fluorescence was observed under an inverted laser confocal microscope (FV1200; New Discovery Technology (China) Co., Ltd., Shanghai, China).

### Western blot

The cells or tumor tissues were split using lysozyme solution (90,082, ThermoFisher, Shanghai, China), and the protein concentration of the cells was measured using a BCA kit (Solarbio, Beijing, China). Then, the protein samples were transferred to sodium dodecyl sulphate-polyacrylamide gel electrophoresis (SDS-PAGE) electrophoresis (Mini-Protean-3, Bio-Rad, Hercules, CA, USA) and transferred onto a polyvinylidene difluoride (PVDF) membrane (Millipore, Massachusetts, USA). After the membranes were blocked with 5% skim milk, they were incubated with primary rabbit anti-human antibodies against β-catenin (1:2000, ab16051, Abcam), CyclinD1 (1:200, ab16663, Abcam), GSK-3β (1:5000, ab32391, Abcam), p-GSK-3β (1:1000, ab131097, Abcam), and β-actin(1:2500, ab8227, Abcam, UK) and mouse anti-human FUT4 (1:1000, sc-19,648, Santa Cruz Biotechnology, Beijing, China). After three washes with TBST (TBS, 1 ml/L Tween-20), the membranes were incubated with horseradish peroxidase-conjugated goat anti-rabbit (1:2000, ab6721, Abcam) and goat anti-mouse immunoglobulin G secondary antibodies (1:2000, sc-2354, Santa Cruz Biotechnology). Finally, the enhanced chemiluminescence (ECL) method was used for detecting signals, and greyscale scanning and quantification of the protein bands were performed by ImageJ (NIH) software 6.0. The expression levels of proteins were normalized to β-actin.

### Animals

Thirty SPF grade BALB/C female nude mice, body weight 16–18 g, 4 weeks old, were purchased from Beijing Weitong Lihua Experimental Animal Technology Co., Ltd. (license no. scxk (Jing) 20,160,006). The animals were raised at 26–28 °C and a humidity of 40–60%. The feed, drinking water and bedding materials were sterilized. Animal experiments followed the national institutes of health guidelines (NIH pub. no. 85–23, revised 1996) and were approved by the Animal Protection and Use Committee of Shengjing Hospital.

### Xenograft tumour model

Thirty mice were randomly divided into 5 groups (*n* = 6): the model group: mice were subcutaneously injected with 200 μL of normal saline; the miR-200c group: mice were subcutaneously injected with 200 μL (5 × 10^6^ cells/100 μL) of LoVo and SW480 cells [16], which were transfected with miR-200c mimic; the si-FUT4 group: mice were subcutaneously injected with 200 μL (5 × 106 cells/100 μL) of LoVo and SW480 cells, which were transfected with siRNA FUT4 lentiviral vector; the miR-200c + NC1 group: mice were subcutaneously injected with 200 μL (5 × 106 cells/100 μL) of LoVo and SW480 cells, which were transfected with miR-200c mimic and pcDNA3.1 empty vector; the miR-200c + FUT4 group: mice were subcutaneously injected with 200 μL (5 × 106 cells/100 μL) of LoVo and SW480 cells, which were simultaneously transfected with miR-200c mimic and pcDNA3.1 FUT4 plasmid.

### Tumour volume

The long diameter (L) and short diameter (W) of the tumour were measured every 7 days, and the tumour volume was calculated. Tumour volume (V) = (long diameter × short diameter ^2^)/2. After 28 days, the nude mice were anaesthetized by intraperitoneal injection of 3% pentobarbital sodium (40 mg/kg) and then sacrificed by cervical dislocation. The tumour tissues were weighed. The positive expression of Ki-67 was detected by immunohistochemistry and immunofluorescence staining.

### Immunohistochemistry

The tumour tissue was heated, dewaxed with xylene, and then hydrated with gradient ethanol solution. A 3% H2O2 methanol solution was added for inactivation for 20 min, high temperature antigen in citrate buffer solution (pH 6.0) was used for thermal repair for 10 min, and 5% BSA was used for blocking treatment for 20 min. Rabbit anti-human Ki67 (1:200, ab15580, Abcam) polyclonal antibody was added and incubated overnight at 4 °C. After rewarming, goat anti-rabbit IgG labelled with horseradish peroxidase (1:1000, abin101988, Antibodies Online, Germany) was incubated with the secondary antibody, and DAB staining was performed. The cells were observed under an optical microscope at 400× magnification (Olympus, Japan). The results are expressed as the percentage of positive cells (%).

### Statistical analysis

SPSS 19.0 statistical analysis software was used for data processing, and the results of data analysis are expressed as the mean ± standard deviation (mean ± SD). The t-test was used for data analysis between two groups, and one-way analysis of variance (ANOVA) with Turkey’s t test was used for data analysis of multiple-group comparisons. The difference was statistically significant at *p* < 0.05.

## Results

### Low expression of miR-200c and high expression of FUT4 in colon cancer cells

The mRNA expression of miR-200c and FUT4 in cells was measured by RT-qPCR. As shown in Fig. 1, the expression of miR-200c mRNA in LoVo (Fig. 1a) and SW480 (Fig. 1b) cells was significantly lower than that in NCM460 cells (*p* < 0.05), and the expression of FUT4 mRNA in LoVo (Fig. 1a) and SW480 (Fig. 1b) cells was significantly higher than that in NCM460 cells (*p* < 0.05). Pearson correlation analysis (Fig. 1c) showed a negative correlation between the mRNA expression of miR-200c and FUT4 (*r* = − 0.9046 for LoVo cells and *r* = − 0.9236 for SW480 cells).

**Fig. 1:** The mRNA expression of miR-200c and FUT4 in colon cancer cells. **a** The mRNA expression of miR-200c and FUT4 in LoVo cells was analysed by RT-qPCR; **b** The mRNA expression of miR-200c and FUT4 in SW480 cells was analysed by RT-qPCR; **c** The correlation between miR-200c and FUT4 in LoVo and SW480 cells was determined using Pearson correlation analysis. Data are expressed as the mean ± SD. The t-test was used for data analysis between two groups. In this experiment, the analyses were repeated 3 times. The resolution of figure is 300 pixels

### FUT4 is a target gene of miR-200c in colon cancer cells

To determine whether FUT4 is a target gene of miR-200 in colon cancer cells, we performed target gene prediction between miR-200c and FUT4 using TargetScan software (www.targetscan.org). As shown in Fig. 2a, we identified potential binding sites for the miR-200c and FUT4 genes. To further verify that miR-200c targets FUT4, we used a dual luciferase reporting system (Fig. 2b). The results showed that the miR-200c mimic could reduce the luciferase activity of the wild-type FUT4 3’UTR but did not decrease the luciferase activity of the mutant FUT4 3’UTR (*p* < 0.05). These results identified FUT4 as a direct target gene of miR-200c in colon cancer cells.

**Fig. 2:** FUT4 is a downstream target gene of miR-200c in colon cancer. **a** Sequence alignment between miR-200c and FUT4. The WT binding sites of miR-200c on FUT4 and its mutated binding sequences are shown. **b** Luciferase activity in cells following cotransfection with miR-200c mimic and luciferase reporters containing WT- or mut-FUT4 transcript. In this experiment, the analyses were repeated 3 times. Data are expressed as the mean ± SD. ^*^p < 0.05. The resolution of figure is 300 pixels

### MiR-200c overexpression inhibits the proliferation of colon cancer cells by downregulating FUT4

To determine the roles of miR-200c and FUT4 in colon cancer cells, we transfected miR-200c mimic, si-FUT4 and FUT4 mimic into LoVo and SW480 cells. The mRNA expression of miR-200c and FUT4 in each group was analysed to show the transfection efficiency using RT-qPCR. In LoVo (Fig. 3a) and SW480 (Fig. 3b) cells, the miR-200c mRNA level was significantly higher in the other groups than in the BC group (*p* < 0.05), while FUT4 mRNA expression showed the opposite trend. Compared with that in the miR-200c + NC1 group, the expression of miR-200c mRNA in the miR-200c + FUT4 group was significantly reduced (*p* < 0.05), while FUT4 mRNA was evidently increased (*p* < 0.05). Furthermore, the proliferation of colon cancer cells in each group was measured by CCK-8 (Fig. 3c) and plate colony formation assays (Fig. 3d). Compared with that of the BC group, the optical density value in the other groups was dramatically decreased (*p* < 0.05). Moreover, the optical density value in the miR-200c + FUT4 group was significantly increased compared with that in the miR-200c + NC1 group (*p* < 0.05). Similar results were obtained from the plate colony formation assay (Fig. 3d). The colony formation numbers were obviously decreased in the other groups compared with the BC group (*p* < 0.05), and the colony formation numbers were clearly increased in the miR-200c + FUT4 group compared with the miR-200c + NC1 group (*p* < 0.05). All these findings suggested that overexpression of miR-200c could inhibit the proliferation of colon cancer cells by downregulating FUT4.

**Fig. 3:** MiR-200c overexpression inhibits the proliferation of colon cancer cells by downregulating FUT4. **a** The transfection efficiency of miR-200c and FUT4 in LoVo cells was measured by RT-qPCR; **b** The transfection efficiency of miR-200c and FUT4 in SW480 cells was measured by RT-qPCR; **c** The cell viability was measured by CCK-8 assays; **d** The proliferation of cells was analysed using plate colony formation assays. ^*^p < 0.05 vs. the BC group; ^#^*p* < 0.05 vs. miR-200c; ^&^*p* < 0.05 vs. miR-200c + the NC1 group. Data are expressed as the mean ± SD. ANOVA with Turkey’s t test was used for data analysis among groups. Each group was analysed in triplicate. The resolution of figure is 300 pixels. BC: blank control group; miR-200c: miR-200c overexpression group; si-FUT4: FUT4 silencing group; miR-200c + NC1: miR-200c overexpression and FUT4 negative control group; miR-200c + FUT4: miR-200c overexpression and FUT4 overexpression group

### MiR-200c overexpression inhibits the migration and invasion of colon cancer cells by downregulating FUT4

The invasion and migration of LoVo and SW480 cells were analysed by transwell assays to determine the roles of miR-200c and FUT4 in colon cancer cells. As shown in Fig. 4, the invasion and migration of LoVo and SW480 cells in the other groups were evidently decreased compared with those in the BC group (*p* < 0.05). Furthermore, compared with that in the miR-200c + NC1 group, the invasion and migration of LoVo and SW480 cells in the miR-200c + FUT4 group was significantly increased (*p* < 0.05). These data demonstrated that overexpression of miR-200c could inhibit the migration and invasion of colon cancer cells by downregulating FUT4.

**Fig. 4:** MiR-200c overexpression inhibits the migration and invasion of colon cancer cells by downregulating FUT4. Transwell assays were used to analyse the effect of miR-200c overexpression on the migration and invasion of LoVo cells (**a**) and SW480 cells (**b**). Magnification: × 400. scale = 50 μm ^*^p < 0.05 vs. the BC group; ^#^*p* < 0.05 vs. miR-200c; ^&^*p* < 0.05 vs. the miR-200c + NC1 group. Data are expressed as the mean ± SD. ANOVA with Turkey’s t test was used for data analysis among groups. Each group was analysed in triplicate. The resolution of figure is 300 pixels. BC: blank control group; miR-200c: miR-200c overexpression group; si-FUT4: FUT4 silencing group; miR-200c + NC1: miR-200c overexpression and FUT4 negative control group; miR-200c + FUT4: miR-200c overexpression and FUT4 overexpression group

### MiR-200c overexpression inhibits the expression of Ki67 in colon cancer cells by downregulating FUT4

The expression of Ki-67 in LoVo and SW480 cells was analysed in each group by immunofluorescence (Fig. 5). In Fig. 5, Ki-67 was labelled using green fluorescence (FITC), and nuclei were labelled using blue fluorescence (DAPI). MiR-200c overexpression or silencing of FUT4 significantly inhibited the expression of Ki67 in LoVo and SW480 cells compared with that in the BC group (*p* < 0.05). Furthermore, compared with that in the miR-200c + NC1 group, the expression of Ki67 was significantly increased after cotransfection of miR-200c and FUT4 (*p* < 0.05). The Ki-67 protein level was also analysed by western blot analysis. Similar results are shown in Fig. 6. The results indicated that miR-200c overexpression inhibited the expression of Ki67 in colon cancer cells by downregulating FUT4.

**Fig. 5:** Immunofluorescence was used to analyse the effect of miR-200c overexpression on the expression of Ki67 in colon cancer cells (magnification, × 400, scale = 50 μm). Ki-67 was labelled using green fluorescence (FITC), nuclei were labelled using blue fluorescence (DAPI), and merge indicates the two fluorescence superpositions. ^*^p < 0.05 vs. the BC group; ^#^*p* < 0.05 vs. miR-200c; ^&^*p* < 0.05 vs. the miR-200c + NC1 group. Data are expressed as the mean ± SD. ANOVA with Turkey’s t test was used for data analysis among groups. Each group was analysed in triplicate. The resolution of figure is 300 pixels. BC: blank control group; miR-200c: miR-200c overexpression group; si-FUT4: FUT4 silencing group; miR-200c + NC1: miR-200c overexpression and FUT4 negative control group; miR-200c + FUT4: miR-200c overexpression and FUT4 overexpression group

**Fig. 6:** Western blot analysis was used to detect the effect of miR-200c overexpression on the expression of Wnt/β-catenin-related proteins in LoVo cells (**a**) and SW480 cells (**b**). ^*^p < 0.05 vs. the BC group; ^#^*p* < 0.05 vs. miR-200c; ^&^*p* < 0.05 vs. the miR-200c + NC1 group. p-GSK-3β/GSK-3β: the ratio of phosphorylated GSK-3β (p-GSK-3β) and total GSK-3β. Data are expressed as the mean ± SD. ANOVA with Turkey’s t test was used for data analysis among groups. Each group was analysed in triplicate. The resolution of figure is 300 pixels. BC: blank control group; miR-200c: miR-200c overexpression group; si-FUT4: FUT4 silencing group; miR-200c + NC1: miR-200c overexpression and FUT4 negative control group; miR-200c + FUT4: miR-200c overexpression and FUT4 overexpression group. The full length blots were presented in Supplementary Figure 1

### MiR-200c overexpression inhibits the expression of Wnt/β-catenin-related proteins by downregulating FUT4

To determine the underlying mechanism of miR-200c and FUT4 in colon cancer, we measured the proteins in the Wnt/β-catenin pathway by western blots. Wnt/β-catenin signalling is an important pathway related to cell proliferation, which can be promoted by upregulating cyclinD1 [17]. β-catenin is the key molecule of the pathway, whose level is regulated by glycogen synthase kinase-3β (GSK-3β) [15]. Figure 6 showed the expression of FUT4, β-catenin, CyclinD1, phosphorylated GSK-3β (p-GSK-3β) and total GSK-3β in each group of LoVo and SW480 cells. Compared with those of the BC group, the levels of FUT4, β-catenin, CyclinD1, and p-GSK-3β were significantly downregulated in the other groups (*p* < 0.05). For the miR-200c + FUT4 group, simultaneous treatment with miR-200c and FUT4 upregulated the expression of the above proteins compared to that of the miR-200c + NC1 group (*p* < 0.05), which indicated that miR-200c overexpression inhibits the expression of Wnt/β-catenin-related proteins by downregulating FUT4.

### MiR-200c overexpression inhibits tumour growth by downregulating FUT4

A xenograft tumour model was established to verify the results in vitro. In vivo*,* the tumour volume (Fig. 7a), tumour weight (Fig. 7b), tumour images (Fig. 7c) and Ki-67 expression (Fig. 7d) were observed to study the effect of miR-200c and FUT4 on tumour growth. Compared with the model group, tumour growth was significantly inhibited in the other groups (*p* < 0.05). Consistent with the in vitro results, tumour growth was clearly increased in the miR-200C + FUT4 group compared with the miR-200C + NC1 group (*p* < 0.05, Fig. 7a-c). The expression of Ki-67 in the tumour tissues was analysed by immunohistochemistry (Fig. 7d). The results showed that the Ki-67 levels were obviously decreased in the miR-200C group and si-FUT4 group, but the trend was weakened in the miR-200C + FUT4 group (*p* < 0.05, Fig. 7d). The data suggested that miR-200C overexpression inhibited tumour growth by downregulating FUT4.

**Fig. 7:** MiR-200c overexpression inhibits tumour growth by downregulating FUT4. **a** Tumour volume; **b** tumour weight; **c** tumour image; **d** the expression of Ki-67 was analysed by immunohistochemistry (magnification,× 400, scale = 50 μm). The resolution of figure is 300 pixels. ^*^p < 0.05 vs. the model group; ^#^*p* < 0.05 vs. the miR-200c group; ^&^*p* < 0.05 vs. the miR-200c + NC1 group. Model: blank control group; miR-200c: miR-200c overexpression group; si-FUT4: FUT4 silencing group; miR-200c + NC1: miR-200c overexpression and FUT4 negative control group; miR-200c + FUT4: miR-200c overexpression and FUT4 overexpression group

### MiR-200c overexpression inhibits the Wnt/nt//0c overexpressby downregulating FUT4 in vivo

The expression of Ki-67, FUT4, β-catenin, CyclinD1, and p-GSK-3β/GSK-3β was also analysed in the tumour tissues by western blots. As shown in Fig. 8, compared with those in the model group, the above proteins in the miR-200c group and si-FUT4 group were significantly decreased (*p* < 0.05). Moreover, treatment with miR-200c and FUT4 evidently increased the expression of the above proteins compared with those in the miR-200c + NC1 group (*p* < 0.05), which indicated that miR-200c overexpression inhibits the expression of Wnt/β-catenin-related proteins by downregulating FUT4 in vivo.

**Fig. 8:** MiR-200C overexpression inhibits the Wnt/β-catenin pathway by downregulating FUT4 in tumour tissues. **a** Wnt/β-catenin pathway-related proteins in LoVo tumour tissues of mice; **b** Wnt/β-catenin pathway-related proteins in SW80 tumour tissues of mice. The resolution of figure is 300 pixels. ^*^p < 0.05 vs. the model group; ^#^*p* < 0.05 vs. the miR-200c group; ^&^*p* < 0.05 vs. the miR-200c + NC1 group. Model: blank control group; miR-200c: miR-200c overexpression group; si-FUT4: FUT4 silencing group; miR-200c + NC1: miR-200c overexpression and FUT4 negative control group; miR-200c + FUT4: miR-200c overexpression and FUT4 overexpression group. The full length blots were presented in Supplementary Figure 2

## Discussion

The biological function of miR-200c in human colorectal cancer remains controversial. Roh MS et al. found that miR-200c was upregulated in 109 paired colorectal cancer patients and increased in colorectal cancer with a higher grade, advanced stage and lymphovascular invasion [18]. Yu et al. [19] reviewed the prognostic value of the miR-200 family in 1882 patients with colorectal cancer showing that high expression of miR-200c was associated with improved colorectal cancer or was related to poor outcomes of colorectal cancer. In colorectal cancer patients, FUT4 was overexpressed in most metastatic colorectal cancer patients (43%) and associated with higher systemic inflammation and poor outcomes [20].

In the present study, the regulatory mechanism of miR-200c in colon cancer metastasis was evaluated by targeting FUT4. We found that miR-200c expression was substantially lower and FUT4 expression was clearly higher in LoVo and SW480 cells than in NCM460 cells. Furthermore, FUT4 is a target gene of miR-200c in colon cancer cells, which negatively regulates miR-200c. In vitro and in vivo, miR-200c overexpression inhibited the proliferation of LoVo and SW480 cells, and FUT4 silencing suppressed the proliferation of LoVo and SW480 cells. These results indicated that miR-200c plays a positive role and FUT4 plays a negative role in the treatment of colon cancer.

The miR-200 family includes five members: miR-200a, miR-200b, miR-200c, miR-429 and miR-141 [21]. In breast cancer, miR-200b was negatively correlated with FUT4, and miR-200b inhibited the proliferation and invasion of breast cancer cells by downregulating FUT4, which inactivated the PI3K/Akt signalling pathway [22]. The FUT family is a class of glycosyltransferase molecules that are involved in the synthesis of glycoproteins and glycolipid sugar chains on the cell surface, which play important roles in a variety of physiological processes [23]. FUT4 has been observed in many cancers, such as breast cancer [22] and colon cancer [20]. In the present study, CCK-8 and plate colony formation assays confirmed that miR-200c overexpression could inhibit the proliferation of LoVo and SW480 cells by targeting FUT4. Furthermore, transwell and immunofluorescence assays suggested that miR-200c overexpression could inhibit the invasion and migration of LoVo and SW480 cells by targeting FUT4. In vivo*,* immunohistochemistry demonstrated that miR-200c overexpression suppressed tumour growth by targeting FUT4.

The Wnt signalling pathway is widely present in invertebrates and vertebrates and is a class of highly conserved signalling pathways during species evolution [12]. A number of studies have shown that the Wnt/β-catenin signalling pathway is associated with a wide variety of human diseases, and miR-200c can inhibit tumour cell migration and invasion by inhibiting Wnt/β-catenin signalling [14, 15]. In acute myeloid leukaemia, silencing FUT4 enhanced the inhibitory effects on p-GSK-3-3β, β-catenin, and CyclinD1 protein expression but not total GSK-3β [24]. Interestingly, the protein expression of β-catenin, CyclinD1, and p-GSK-3β was downregulated after miR-200c overexpression or silencing of FUT4 in this study. However, simultaneous treatment with miR-200c and FUT4 upregulated the expression of the above proteins.

## Conclusions

In conclusion, our study demonstrated that miR-200c was expressed at low levels in colon cancer. In vitro and in vivo, this study also emphasized that miR-200c targets FUT4 to suppress proliferation and migration by inhibiting Wnt/β-catenin signalling. Our current study highlights candidates for gene therapy for colon cancer through miR-200c/FUT4.

## Supplementary Information

**Additional file 1: Supplementary Figure 1**. The original blots of Ki-67, FUT4, β-catenin, Cyclin D1, p-GSK-3β, GSK-3β in Lovo and SW480 cells. (Corresponding to Fig. 6 in the manuscript).

**Additional file 2: Supplementary Figure 2.** The original blots of Ki-67, FUT4, β-catenin, Cyclin D1, p-GSK-3β, GSK-3β in Lovo and SW480 cells. (Corresponding to Fig. 8 in the manuscript).

## Data Availability

The datasets used and/or analysed during the current study are available from the corresponding author on reasonable request.

## Abbreviations

FUT4: Fucosyltransferase 4
RT-qPCR: Real-time quantitative polymerase chain reaction
CCK-8: Cell counting kit-8
CRC: Colorectal cancer cells
FBS: Foetal bovine serum
BSA: Bovine serum albumin
PBS: Phosphate-buffered saline
DAPI: 4′,6-diamidino-2-phenylindole
SDS-PAGE: Sodium dodecyl sulphate-polyacrylamide gel electrophoresis
PDVF: Polyvinylidene difluoride
ECL: Chemiluminescence
ANOVA: One-way analysis of variance (ANOVA)
GSK-3β: Glycogen synthase kinase-3β
